RETRACTED

# College Physical Education and Training in Big Data: A Big Data Mining and Analysis System

**DOI:** 10.1155/2021/3585630

**Published:** 2021-11-30

**Authors:** Huiqin Wang

**Affiliations:** Nanyang Medical College, Nanyang, Henan 473061, China

## Abstract

Recently, big data has been broadly used as a research method in all aspects of analysis, prediction, and evaluation. The application of big data to college students' physical education plays a significant role in encouraging the completion of physical education at various levels. The application of the Internet and the advent of smartphones impact the way college students participate in physical exercise. At present, more and more students begin to participate in sports, and students' demand for physical training is increasing. During physical education training, a lot of data is generated every moment because of various actions and behaviors. Due to technical limitations, these data were not effectively collected and applied. In this environment, the development and management of sports data mining systems have become more and more important. This paper designs an intelligent big data system for college physical education training. The study mainly focuses on data decentralization, lack of data talents, insufficient technical support, and low utilization of venues in physical education. While designing a big data system, the data is collected based on ease of data collection, and a response framework with excellent performance in storing analytical data is selected. The design and management of this system have a certain significance for the improvement and optimization of current college physical education training.

## 1. Introduction

Artificial intelligence and big data techniques are increasingly penetrating into all walks of life. Big data has quickly and accurately occupied the desks of workers in various industries. The use of big data and artificial intelligence in the college physical education industry has brought certain challenges and opportunities to the traditional higher education industry. Big data is both a resource and a research method [1].

Recently, the application and importance of data mining have been realized. In competitive sports, data mining methods have been employed in specialized information statistical analysis [2]. Data mining is a type of information processing technique that combines several technologies and related models such as information technology, pattern recognition, mathematical statistics, machine learning, and data visualization. It can assist the extraction of information that is potentially valuable and facilitate the effective utilization of potential information. It collects and analyzes the hidden data and stores the valuable data [3]. Data mining transforms everyday behavior and information into data, transforms data into mathematical models, converts logical conclusions into knowledge, and applies knowledge to decision making and action. Moreover, data mining technology is a new method that can increase efficiency and scientific decision making. The information extracted by data mining has the features of validity, practicability, and unknowingness [4].

RETRACTED

The development of college sports is an important link in the development of sports. Many scholars have conducted comprehensive research on the assessment of college physical education using big data. Xiong [5] explored the application of big data to physical education and reported that the creation of physical education big data platform helps advance the physical education informatization, the development of modern talents, and finally the development of higher level education. Paper et al. [6] argued that multimedia education can increase college students' interest in learning in physical education, can help uncover the important and difficult points in physical education, and can contribute to the understanding of proper coordination. Liu and Bu [7] applied the grey GM prediction model and used questionnaire approach to build an online education platform and develop an effective education model method, to combine the best educational resources and ease time and space constraints in learning physical education. The method was used to provide a relaxing learning environment for physical education, where one can learn anytime, anywhere. Liu et al. [8] proposed to form a physical education teaching system and supplement the physical education action plan to improve the content, form, and method of physical education teaching. Lee and Hokanson [9] showed that contribution to extracurricular sports events has a constructive impact on the academic performance of higher education students; that is, participation in regular sports events has a strong relationship with the college students' scores.

Hu and Ye [10] studied the application of big data to find the diversity of teaching in physical education. The final result reported that big data has a great impact on the investigation of diversity in the teaching of physical education. Compared with conventional physical education content, it not only improves students' interest in learning but also increases the physical fitness of students. However, their investigation was based on few data samples, and the accuracy of the data was very low. Jane et al. [11] have completed thorough research on big data and physical education and obtained very excellent results. However, with the fast growth of computers, this research has become increasingly impotent to meet the needs of college students.

RETRACTED

With the progress of video and image processing techniques, it is usual to apply video analysis techniques to sports analysis scenarios. The author in [12] used several cameras to record the entire field of a soccer match, to capture the on-field actions and paths of each player. For this purpose, a system is proposed to get the track of the paths, actions, and trajectories of each player during a match. The algorithm can detect the targets by creating individual models based on topographies and athletes' motion trends and can help coaches statistically investigate and analyze the tactical runs and behavior of athletes during the match. A human fitting model using morphological methods in a simple context was proposed by Li et al. [13]. The method was effective in locating the four key joints of the body and extracting the angular statistics of the body to assist the players in correcting their daily physical training. The object of this study is to solve the problem of data dispersion in the practice of college sports, the cultivation of physical education talents, and the low utilization rate of venues and to provide an efficient way to solve problems through big data systems. A universal data system is established; it is easy to use, helpful in teaching students following their aptitude, and conducive to continuously improving the teaching level and strengthens the management and operation of physical education in colleges and universities.

The rest of the paper is ordered as follows: In Section 2 different shortcomings and aspects of the college physical education system are described. In Section 3 the framework of the proposed college physical education system is explained, and finally the conclusion is given in Section 4.

## 2. Data Dilemma of College Physical Education

### 2.1. Decentralization of Data in College Physical Education

Because of the simplicity of the data types and the ease with which data is collected, subsequent analysis and storage of the data are relatively straightforward. However, the generation and collection of physical education data in colleges and universities are not so simple [14]. The data of college physical education not only includes the students' performance in the class and the mastery of the theory but also reflects the students' daily sports and the physical data of the students themselves. In general, college physical education teaching data can be collected mainly from sports health test data, sports meeting data, sports theory score data, course number data, exercise time-frequency data, and physical quality data. The data sources of college physical education are shown in Figure 1.

RETRACTED

Sports health data is the data generated by the annual “sports assessment”, an important activity of colleges and universities. Sports data is the best data to measure the effect of students' exercise. The sports theory data is the horizontal display of students' sports level and physical education level data. The course number data facilitates the aggregation and calculation of data such as the total amount and average value of sports data. The time and frequency data of exercise show the enthusiasm of the individual for sports and the effect of sports on the individual to help the teacher to develop a personalized teaching plan. The physical quality data is a comprehensive evaluation of the physical quality of the students themselves from an objective perspective. The development of college sports has made some progress today, such as using the Internet in teaching and using apps to improve students' interest in learning. However, there are still some shortcomings [15]. These problems can be solved through big data. To realize the high efficiency of physical education in colleges and universities, keeping in mind the current shortage of teaching resources and outdated teaching strategies in college physical education, this paper proposes the application of technology and information of big data to reform college physical education in the context of “big data” and promote the development of college physical education.

### 2.2. Lack of Data Talents in Physical Education

Faced with the advancement of technology and the development of the industry, the lack of talent has become the common voice of all fields of life, especially in the big data industry. Big data and artificial intelligence have been covered in various industries [16]. This huge talent gap covers all enterprises and institutions that want to be the leader in the era of intelligent technology. To cope with the development of the big data era, in addition to actively opening big data courses, colleges and universities are also very important manifestations of big data applications in teaching work. The lack of big data talents in the entire industry is also reflected in college physical education.  Figure 2 shows the statistical data of talents' ability in college sports data.

According to statistics, the skills required for college physical education data talents include data processing, data modeling, report writing, data delay, data monitoring, data forecasting, decision-making recommendations, and special analysis. Simple data analysis itself does not make sense, and data analysis is not as complicated as believed. A target dataset is used for data analysis, trying to explore the meaning behind the data and the role of the data itself, and any behavior and information in physical education training can be digitized. The ultimate goal of data analysis is to complete the decision-making optimization and improvement of physical education training. The need for physical education data talents requires mastering not only the basic data analysis skills but also the basic principles and basic laws of college physical education. The output of analytical results is also necessary. In recent years, physical education in colleges and universities has made significant progress in curriculum construction, students' participation in physical exercise, improvement of scientific research level, and relevant conditions. It has laid a foundation for improving students' physical health, promoting higher education reform, and improving education quality. However, there are still many difficulties and problems in the physical education of colleges and universities [17].

RETRACTED

In general, due to the lack of necessary basic systems, standards, and clear requirements, the gaps in sports work between regions and schools are large, which affects higher education institutions. On the whole, the decline in the physical health level of college students has not been fundamentally reversed. It is the basic requirement for the physical education of full-time ordinary colleges and universities. It is an important metric for measuring the physical education of colleges and universities. In addition to the specific skills of sports data processing and data modeling, data monitoring, data prediction, and special analysis are also important skills. In the selection and training of data talents, attention must be paid to the comprehensive ability of sports data talents.

### 2.3. Rigidity of Physical Education System

The main purpose of college education in China is to carry out professional education to promote professional specific talents after completing secondary education. For this purpose, physical education in colleges and universities is often carried out as an auxiliary subject, but in theory, physical education is a very important activity in the social subconscious. At present, there are problems in the entire university education system, such as the lag of the enrolment training system, the lag of the university teaching management system, and the lag of the discipline setting. It is also reflected in the college physical education system. The system structure of physical education in colleges and universities is shown in Figure 3.

RETRACTED

In addition to a small number of students majoring in physical education, the physical education system of college students is to set up a physical education department under the unified management of the school's education department. Under the physical education department, the teaching department, research department, and management department are separately set up [18]. It can be seen from the department settings that the department settings are scattered, and the data between departments is not easy to communicate, resulting in the phenomenon of data islands. The Ministry of Physical Education and the teaching and research section should regard teaching and education as an important part of the teacher's teaching evaluation and business assessment. The evaluation and assessment data are stored in the teacher's business file, which is an important basis for promotion and appointment. This causes us to have many inconveniences when using technical means to solve the problem of physical education. The technical means cannot be used to solve the problems set by the sports department. Because of the problems of department setting and management, there is no technical personnel involved [19]. The circulation of data flow in this is not smooth enough, and problems cannot be solved in time. On the other hand, in response to the surging information and data era, the choice of the physical education department is to turn a blind eye and not to take into account the technical problems of the department.

### 2.4. Inadequate Use of University Sports Venue Data

One of the main reasons for the limited development of sports in China is the strong demand for sports and the lack of social sports resources. This is particularly evident in the process of physical education in colleges and universities. Due to the high maintenance cost of sports venues and the relatively tight funding for running colleges and universities, many colleges and universities have abandoned the construction and maintenance of sports venues, resulting in some colleges and universities not having sufficient teaching venues, but the colleges and universities with venues have not been properly maintained and used, resulting in lack of resources. The influencing factors of university stadiums are shown in Figure 4.

To avoid the wastage of existing venues in colleges and universities, the utilization data of existing venues should be collected, and feedback should be provided. The main factors affecting the use of college venues include security factors, class time, management system, operational mechanism, economic conditions, and distance factors [20]. Effective collection and analysis of these data and intuitive display of the use of the venue can play a role in the rational use of the venue. Safety factors are the primary issues to be considered during the use of the venue. The unsafe training environment will directly affect the credibility of the venue and whether data can be collected. Class time is also a special influencing factor in the university environment. The primary function of college venues is teaching. When intelligent big data systems are designed, the index of this factor needs to be higher. The management system and operational mechanism will be related to the open time and form of the venue. The efficient and reasonable open form is a necessary condition for the effective use of the venue resources. Under the current education system, the local economic conditions and the economic conditions of the university are the core factors affecting the construction of the field. The distance factor is also a problem that needs to be measured. When designing big data systems, the proportion and sequence of the above factors are issues that need to be considered.

RETRACTED

## 3. Methodology

### 3.1. The Framework of College Physical Education Teaching Data System

In the construction of college sports education big data system, the requirements that need to be completed included the construction of data collection platform, the stratification of student behavior data warehouse, the construction of data warehouse of college sports venues, and the efficient storage and reading. In the technology selection, the Hadoop file system was used; it includes component such as HDFS (Hadoop Distributed File System), MapReduce, YARN, HBase, Pig, Hive, Sqoop, Flume, Kafka, ZooKeeper, and Spark. The big data system of college physical education is shown in Figure 5.

Even with big data architecture, the application layer is still a traditional web application, but it will store data according to the characteristics of the data (structured data will still be stored in traditional relational databases such as MySQL; nonstructural data such as logs will be saved in a distributed file system such as HDFS for Hadoop). Big data is an enhancement to web applications. Based on distributed storage and distributed computing, the problems that were previously unsolvable by stand-alone or small-scale clusters can be solved by using big data technology, such as logs and other data when the amount of data is very large (terabytes or even petabytes). The analysis of such a large amount of data is impossible or very slow on the traditional architecture. It is possible to use the big data technology mainly for dividing the data processing on different nodes (computers) through MapReduce, then merge the results, and generate final analysis [21].

RETRACTED

The main related framework features and functions of Hadoop are as follows: HDFS is a widely used distributed file system, which is the basic general file storage component of the entire big data application scenario. MapReduce is the basic computing framework for distributed computing. HBase is a NoSQL column family database and supports billions of rows and millions of columns of large data storage and access, especially in scenarios where data performance is time sensitive. It does not support SQL queries. Hive uses SQL for statistics and analysis to generate query results. The component can be used to generate tasks performed on the MR by parsing HQL. The typical application scenario is integrated with HBase. Hive is a data warehousing tool and can be seen as a user programming interface to some extent. It does not store and process data itself; instead, it relies on HDFS to store data and relies on MapReduce to process data. Hive defines a simple SQL-like query language, HiveQL, which is compatible with most SQL syntaxes. However, it does not fully support SQL standards. For example, HiveQL does not support update operations, nor does it support indexes and transactions. There are also many limitations to the connection operation. HiveQL statements can quickly implement simple MapReduce tasks, so users can run MapReduce tasks by writing HiveQL statements without having to write complex MapReduce applications. For Java development engineers, it is not necessary to spend a lot of effort memorizing the correspondence between common data operations and the underlying MapReduce Java API [22]. For database administrators (DBA), it is easy to port the data warehouse application originally built on a relational database. Hive is an analysis tool that can organize and use data efficiently, reasonably, and intuitively. Kafka is a distributed, subscription-based messaging system, similar to the function of message queue, which can accept producers. The data itself can be cached and then sent to the consumer for buffer adaptation. Flume is a distributed system for massive log collection, aggregation, and transmission; the main function is the collection and transmission of data, and it also supports more input and output data sources.

### 3.2. Adaptive Learning Algorithm for College Physical Education

The adaptive process is a process of constantly approaching the goal. The approach it follows is represented by a mathematical model called an adaptive algorithm. Gradient-based algorithms are commonly used, with the least mean square error algorithm (LMSE algorithm) being especially common [23]. The adaptive algorithm can be implemented in either hardware (processing circuit) or software (program control). The former designs the circuit according to the mathematical model of the algorithm, while the latter formulates the mathematical model of the algorithm into a program and implements it with a computer. The choice of the algorithm determines the performance quality and feasibility of the processing system.

RETRACTED

The optimal criteria used by the adaptive algorithm are the least mean square error (LMSE) criteria, least squares (LS) criteria, maximum signal to noise ratio (SNR) criteria, and statistical detection criteria [24]. The multiplication criterion is currently the most popular adaptive algorithm criterion. It can be seen that the LMSE algorithm and the RLS algorithm have different optimal criteria, so the two algorithms have many differences in performance and complexity.

(1) $$\begin{array}{c} p\left(x\right)=p_{n}\left(x\right)=\sum_{j=0}^{n}c_{j}x^{j}. \end{array}$$

The coefficients of the polynomial are not directly related to the given data points; therefore, the polynomial basis function is added, and such an expression is very easy to operate, for different points or interpolation formulas. The calculation process can be designed in this way during the actual calculation process. According to the distance from the interpolation point *x*, the interpolation nodes *x*_0_, *x*_1_,…, *x*_*n*_ are arranged in order; then, a stepwise interpolation table is generated row by row; and a new node is introduced for each additional row until the deviation of the two diagonal elements meets the accuracy requirements. This is the adaptive method of stepwise interpolation.

(2) $$\begin{array}{c} j\left(n\right)=E{\left[e\left(n\right)\right]}^{2}. \end{array}$$

This is the objective function of the algorithm. The least squares method can be seen as another representation of the Wiener filter theory. The Wiener filter is derived from a set of averages, and the least squares method involves the use of time averaging, so the filter depends on the number of samples that are applicable in the calculation. The RLS algorithm calculates the data using the least squares estimate of the filter weight vector at *n* − 1.

The amount of data on Internet learning parameters is extremely large, and the accumulated data over time is still proliferating; machine learning techniques may be of great help in solving big data processing, which may save significant time and labor costs. At the same time, machine learning optimizes the performance of computer programs by using data or experience. In human learning or people's online learning, the system platform is based on machine learning technology. In terms of machine learning, adaptive learning is only a semi-intelligent personalized learning guide through data processing and fixed algorithms.

RETRACTED

### 3.3. Work Flow of College Physical Education Teaching Data System

Big data refers to the big data generated by the interaction and integration of things, people, and machines in cyberspace and can be obtained on the Internet. For the problems mentioned in Section 2, the proposed system solves the problem by collecting, analyzing, and displaying the data. First of all, the students' scattered data is collected through Flume and Kafka, using the terminal's app. This data collection method is used to improve the economic conditions, and now the college students are per capita terminal equipment. In addition to mobile phones, computers, and other clients, there are portable devices such as wristbands that collect students' data in a comprehensive way. Second, given the lack of data talents in college physical education, this system mainly considers the solution through teaching and training and stores a large amount of training data in HDFS. The HBase stores the link address of these data with Hive for query through the terminal interface and transfers data to the user for viewing and learning. When training university physical education talents, some simple teaching content can be directly taught in this way. Third, because of the rigidity of the university system and the inconvenience of information technology joining and maintenance, the system uses the micro-service approach to split the logic of collecting data and analyze the data in the teaching process through the Spring Boot framework. Finally, for the venue usage problem, the Mahout framework is adopted here, through a large amount of historical data, real-time monitoring, and design of the venue's usage plan to ensure the use rate of the venue and avoid waste of resources. The details of data flow platform are given in Table 1.

When performing stream data processing, it is necessary to consume the upstream data source and output the data to the specified storage after processing the data for later data analysis. This process is a data flow; then, the design elements responsible for participating in it can be called the data flow model.

In the past, data synchronization was divided into full-scale synchronization and incremental synchronization, and full-scale synchronization was based on batch processing. However, in the case of big data, a batch will take a long time. The longer the time is, the more difficult it is to ensure reliability, so there is a broken situation. Data Pipeline can solve this problem by managing the position of the data transmission to make the breakpoint resume. When a large-scale data task is to be completed, even if there is data failure, the point can be broken to continue the previous task, reduce synchronization time, and improve synchronization efficiency.

RETRACTED

When synchronizing multiple tasks, it is difficult to balance the pressure of the data transmission to the destination. The transmission under large data volume can be especially reflected. At this time, Data Pipeline can be used to accomplish multiple related tests to optimize different ones. The connection pool can be used to customize open data transmission, customize the appropriate transmission tasks for their business systems, and optimize and adjust the transmission of different kinds of databases to ensure the efficiency of data transmission. In conventional database system support for heterogeneous data, types are not always flexible, and the types are not complete. With the high precision of data in the financial field, the loss of precision caused by the transmission of traditional databases to big data platforms is a big problem. Data Pipeline supports this with more data types, such as the complex types supported by Hive, as well as decimal and timestamp types.

The maintenance of big data systems is also very important. ZooKeeper's cluster configuration can be used in the maintenance process. During the maintenance of the cluster, ZooKeeper can efficiently view the status of each node in the cluster and establish a high availability mechanism to ensure efficient and smooth operation of the big data system, without increasing the number of users or increasing the amount of data. There are problems such as downtime. With the big data system, the reasonable use of the system is also a problem that must be considered. When using it, college educators and students need to establish contact between the system and themselves as soon as possible to learn from each other's characteristics and habits. Using the above methods, the use of big data systems can be used to help college physical education training better.

## 4. Conclusion

The collection and analysis of human motion data constitute an indispensable process in the analysis of all sports. With more and more people taking part in sports, digital technology is increasingly involved in sports of sports enthusiasts. Data is the most precious resource, and big data technology has become the focus of cooperation among all walks of life. Sports are one of them. Nowadays, in all kinds of high-profile professional sports competitions, big data is becoming another venue outside the arena. Faced with the problem of data dispersal in physical education, lack of data talents, limited physical education system, and inability to update the information of venues, this paper designed a big data system, through its performance and business logic. The study mainly focuses on data decentralization, lack of data talents, insufficient technical support, and low utilization of venues in physical education. The data is collected based on ease of data collection, and a response framework with excellent performance in storing analytical data is selected. The development and management of this system have a certain significance for the design and optimization of current college physical education training.

RETRACTED

## Figures and Tables

**Figure 1:** Data sources of physical education in colleges and universities.

**Figure 2:** College physical education data talent ability.

**Figure 3:** College physical education institution.

**Figure 4:** Influencing factors of college sports venues.

**Figure 5:** College sports teaching big data system.

**Table 1:** Details of data flow platform.

Platform	Data abstraction	Data flow	Delay	Resource management	Autoscaling
Flume	Event	Agent	Low	Native	No
NiFi	FlowFile	Flow	Configurable	Native	No
Gearpump	Message	Streaming application	Very low	YARN	No
Apex	Tuple	Process topology	Very low	YARN	Yes
Kafka streams	Kafka stream	Application	Very low	YARN	No
Spark streaming	DStream	Topology	Medium	YARN	Yes
Storm	Tuple	Job	Very low	YARN	No
Samza	Message	Streaming data flow	Low	YARN	No
Flink	DataStream	Job	Very low	YARN	No
Ignite streaming	Ignite data streamer	Pipeline	Low	YARN	No
Beam	PCollection	Job	Low	YARN	Yes

## Data Availability

The data used to support the findings of this study are included within the article.
